The article "Dihydroartemisinin targets fibroblast growth factor receptor 1 (FGFR1) to inhibit interleukin 17A (IL-17A)-induced hyperproliferation and inflammation of keratinocytes" was retracted in 2024. Reasons: original data or images not available; concerns about the data; concerns about the results or conclusions.

# Dihydroartemisinin targets fibroblast growth factor receptor 1 (FGFR1) to inhibit interleukin 17A (IL-17A)-induced hyperproliferation and inflammation of keratinocytes

**DOI:** 10.1080/21655979.2021.2021701

**Published:** 2022-01-10

**Authors:** Baojiang Chen, Chen Li, Guizhen Chang, Huan Wang

**Affiliations:** a Department of Dermatology, Tianjin TEDA Hospital, Tianjin, P.R. China; b Department of Internal Medicine, Tianjin Beichen Traditional Chinese Medicine Hospital, Tianjin, P.R. China

**Keywords:** Dihydroartemisinin (DHA), fibroblast growth factor receptor 1 (FGFR1), psoriasis, IL-17A

## Abstract

Psoriasis is a common chronic immune-mediated disease that often has a serious negative impact on the physical and mental health of patients. Dihydroartemisinin (DHA) is a drug with anti-fibrotic and anti-inflammatory effects that may be involved in the autoimmune regulation of immune diseases. However, the effects of DHA on psoriasis have not been reported comprehensively. Therefore, the aim of this study was to investigate the effect of DHA on abnormal proliferation and inflammation of epidermal keratinocyte cells in psoriasis and its mechanism of action. IL-17A-induced human epidermal keratin-forming cells (HaCaT) were used as a model. And after induction exposure to different concentrations of DHA, CCK-8, EDU staining, wound healing and Western blotting were performed to assess cell viability, proliferation, migration, differentiation and inflammatory factors, respectively. Subsequently, agonists of fibroblast growth factor receptor 1 (FGFR1) were added and the above experiments were repeated. The results showed that DHA obviously inhibited IL-17A-induced hyperproliferation, migration and expression of inflammatory factors in HaCaT cells. Furthermore, FGFR1 was highly expressed in IL-17A-induced HaCaT cells, and DHA inhibited its expression. However, the inhibitory effect of DHA on IL-17A-induced HaCaT cells was reversed after the addition of FGFR1 agonist. In conclusion, DHA could inhibit IL-17A-induced hyperproliferation and inflammation of keratinocytes by targeting FGFR1, which also provided a new target for the treatment of psoriasis.

## Introduction

Psoriasis is a common chronic immune-mediated skin and joints disease that often has a negative impact on the physical, emotional and psychological health of patients [1,2]. In approximately 80% of cases, patients with psoriasis showed significant decreases in emotional well-being, ability to function socially, and productivity at school or work [3]. Psoriasis is characterized by persistent inflammation leading to abnormal keratinocyte proliferation and dysfunctional differentiation [4]. Its pathogenesis is complex and multifactorial, and can be generally divided into an initial phase caused by trauma, infection or drugs and a maintenance phase marked by chronic clinical progression [2,4]. Currently, patients with mild psoriasis are mostly treated with topical corticosteroids, vitamin D analogs, calcium-regulated phosphatase inhibitors, keratolytic, and targeted phototherapy [5]. Notably, inflammatory cells in psoriasis released interleukin (IL)-23 and IL-12, which activate IL-17-producing T cells, Th1 cells and Th22 cells, producing large amounts of IL-17, TNF and IL-22 [6,7]. These cytokines might lead to excessive proliferation of keratin-forming cells, which in turn exacerbates psoriatic inflammation. Therefore, it is crucial to study these cytokines and immune disorders in psoriasis research and to improve the therapeutic efficacy of psoriasis by effectively inhibiting the inflammatory response and keratinocyte proliferation.

Dihydroartemisinin (DHA, Figure 1a) is an artemisinin derivative [8]. According to reports, DHA has anti-fibrotic and anti-inflammatory effects and is involved in the regulation of autoimmunity in several immune diseases, such as collagen-induced arthritis, autoimmune thyroiditis and psoriatic skin inflammation [9–11]. Studies have shown that DHA ameliorated psoriasis skin inflammation and inhibits relapse by reducing CD8 + T cell memory in wild-type and humanized mice, attenuated systemic lupus erythematosus by restoring Treg/Th17 homeostasis, and attenuated high glucose-induced vascular smooth muscle cell proliferation and inflammation by inhibiting the miR-376b-3p/KLF15 pathway [11–13]. However, the effect of DHA on the abnormal proliferation of keratinocytes due to psoriasis had not been reported.

**Figure 1.** DHA inhibits over proliferation of IL-17A-stimulated HaCaT cells. (a) The chemical structure of DHA; (b) Cell viability following the different concentration DHA treatment was detected by CCK-8; (c) Cell proliferation was detected with EDU staining; (d) Cell proliferation-related protein expressions were analyzed by Western blotting, including Ki-67, cyclin D1 and c-Myc. **P < 0.01 and ***P < 0.001 vs. control. #P < 0.05, ##P < 0.01 and ###P < 0.001 vs. IL-17A. DHA, dihydroartemisinin.

In the present study, we investigated for the first time the effect of DHA on IL-17A-induced keratinocytes and its potential mechanisms. DHA was predicted to target the fibroblast growth factor receptor 1 (FGFR1) through Swiss Target Prediction database (http://www.swisstargetprediction.ch/). The mechanism was subsequently further validated by examining cell proliferation, migration, differentiation and inflammation.

## Materials and methods

### Cell culture and model

The human epidermal keratinocyte cell line (HaCaT) was provided by the Chinese Academy of Sciences. Cells were grown in RPMI-1640 medium containing 10% FBS and 1% penicillin-streptomycin solution. The culture environment was a standard incubator at 37°C with 5% CO_2_. The incubator contained 5% CO_2_ and was set at 37°C. Cells were defined as the model group (IL-17A group) after 24-hour incubation with 100 ng/mL recombinant human IL-17A (Pepro Tech Inc.) [14].

### Cell vitality assay

Cell viability was determined using Cell Counting Kit-8 (CCK-8) (Beyotime Biotechnology Co., Ltd). Cells were inoculated in 96-well plates (4 × 10^3^ cells/well) and incubated with DHA (3, 10 and 30 μM, respectively) for 24 h at 37°C, followed by addition of CCK-8 solution and incubation for another 2 h at 37°C. The absorbance at 450 nm was measured using an enzyme marker (Bio-Rad Laboratories, Inc.).

### 5-Ethynyl-2’-Deoxyuridine (EDU) staining

Cell proliferation was analyzed by using the BeyoClick™ EdU kit (#C0071S, Beyotime Biotechnology Co., Ltd). Briefly, cells were incubated with EDU labeling solution for 1.5 h at 37°C and then immediately fixed with 4% paraformaldehyde for 15 min at room temperature. Cells were subsequently incubated with 0.5% Triton® X-100 buffer for 20 min at room temperature, and click reaction buffer was added. Finally, the cells were stained with Hoechst for 20 min at room temperature and observed under a fluorescent microscope (magnification, x200).

### Wound healing assay

Cells (3x10^5^ cells/well) were inoculated in 6-well culture plates. After cells were grown to 80–90% confluent, the cells were scratched against with a 20-μl pipette tip and starved. After wound formation, the scratch area was photographed with a light microscope at 0 h and 24 h (magnification, x100). The images were quantified using ImageJ software (version 1.52 r; National Institutes of Health).

### Enzyme-linked immunosorbent assay (ELISA)

Tumor necrosis factor α (TNF-α), IL-1β and IL-6 were quantified by using an ELISA kit (Elabscience Biotechnology Co., Ltd). Briefly, HaCaT cells were seeded in 96-well plates (5x10^3^ cells/well). After 24 h, the cells in different groups were treated for corresponding induction. Subsequently, the cells were centrifuged at 1500 x g with 4°C for 5 min, and the cell supernatants were collected to detect the secretion of inflammatory cytokines according to the ELISA kit instructions.

### Reverse transcription-quantitative PCR (RT-qPCR)

Total RNA was obtained by isolation with Trizol reagent (Invitrogen, Thermo Fisher Scientific, Inc.) according to the manufacturer’s instructions. Reverse transcription was performed using the PrimeScript™ RT Reagent kit (Takara Bio, Inc.). iTaq™ Universal SYBR® Green Supermix (Bio-Rad Laboratories, Inc.) was used to detect FGFR1 expression. Thermal cycling conditions: initial denaturation at 95°C for 10 min; denaturation at 95°C for 15 s and annealing at 60°C for 1 min for 40 cycles; followed by extension at 72°C for 10 min. The following primers pairs were used: FGFR1 forward 5’-CCCGTA GCTCCATATTGGACA-3’ and reverse 5’-TTTGCCATTTTTCAACCAGCG-3’, GAPDH forward 5’-ACAACTTTGGTATCGTGGAAGG-3’ and reverse 5’- GCCATCACGCCACAGTTTC-3’. Relative expression levels were compared using the 2^−ΔΔCq^ method [15].

### Western blotting assay

Cells were disrupted with the lysis buffer. Then, protein content was determined with the BCA protein assay kit. Quantitative protein samples were separated by SDS-PAGE and transferred to polyvinylidene fluoride membranes, which were then closed with 5% skim milk for 1 h at room temperature. Samples were incubated with primary antibody overnight at 4°C and then incubated with secondary antibody for 2 h at room temperature. The signals were visualized using an enhanced chemiluminescence (ECL) kit (Thermo Fisher Scientific, Inc.). Protein expression levels were semi-quantified using Image-Pro Plus version 6.0 (Media Cybernetics, Inc.) software.

### Statistical analysis

All experiments were repeated more than three times. Data were expressed as mean ± standard deviation (SD). GraphPad Prism 8.0 software (GraphPad software, Inc.) was used for statistical analysis. Differences were compared by one-way ANOVA and Tukey’s test. Data are statistically different at P < 0.05.

## Results

### DHA inhibits excessive proliferation of IL-17A-stimulated HaCaT cells

Cell proliferation was detected by using CCK-8 and EDU staining (Figure 1b,c). The results showed that the IL-17A stimulation caused a significant increase in cell viability compared to the control group (Figure 1b), and the EDU staining results indicated that IL-17A stimulation caused excessive cell proliferation (Figure 1c). In contrast, IL-17A-stimulated cell overproliferation became dose-dependently reduced with increasing DHA (Figure 1c). Proliferation-related protein expression was analyzed by Western blotting assay (Figure 1d). The results demonstrated that Ki-67 protein expression was significantly increased following cell stimulation with IL-17A compared to the control group. After the addition of DHA, Ki-67 expression decreased dose-dependently with DHA compared to IL-17A stimulation alone. In addition, the protein expression trends of cyclin D1 and c-Myc were consistent with that of Ki-67 affected by IL-17A and DHA. Therefore, it indicated that DHA could inhibit IL-17A-induced cell over-proliferation.

### DHA inhibits migration, induces cell differentiation and reduces inflammatory response in IL-17A-stimulated HaCaT cells

Migration of IL-7A-induced HaCaT cells was analyzed by wound healing and Western blot (Figure 2a,b). The results showed that induction of IL-17A alone significantly increased the cell migration compared to control group (Figure 2a), and the expression of migration-associated proteins MMP2 and MMP9 were also significantly increased (Figure 2b). In contrast, compared to the IL-17A group, cell migration was inhibited with increasing doses of DHA (Figure 2a), and the expression of related proteins MMP2 and MMP9 were decreased in a dose-dependent manner (Figure 2b). To further investigate the HaCaT cell differentiation, the expression of Keratin 1 and other cell differentiation-related proteins were detected by Western blot (Figure 2c). The results showed that the protein expression of keratin 1, keratin 10, involucrin and filaggrin were significantly inhibited by IL-17A stimulation. However, the protein expression of keratin 1 subsequently increased with DHA dose, and the same trend was observed for keratin 10, involucrin and filaggrin. In addition, RT-qPCR and ELISA were performed to detect inflammatory responses in HaCaT cells (Figure 3a,b). The inflammatory factor expressions were significantly increased in cells stimulated by IL-17A compared to control group. Nevertheless, the expressions of TNF-α, IL-1β and IL-6 in cells were remarkably suppressed in the presence of DHA with a dose-dependent trend. Notably, the detection of inflammatory response-related pathway protein expressions found that IL-17A significantly induced the inflammatory response, in contrast, DHA significantly inhibited the inflammatory response (Figure 3c). Taken together, these results suggested that DHA not only inhibited the migration of IL-17A-stimulated HaCaT cells, but also promoted the differentiation and attenuated inflammatory response such cells.

**Figure 2.** DHA inhibits migration and induces cell differentiation in IL-17A-stimulated HaCaT cells. (a) Cell migration was detected by using wound healing; (b) Cell migration-related protein expressions were analyzed by Western blotting, including MMP2 and MMP9; (c) Cell differentiation-related protein expressions were analyzed by Western blotting, including keratin1, keratin 10, involucrin and filaggrin. ***P < 0.001 vs. control. #P < 0.05, ##P < 0.01 and ###P < 0.001 vs. IL-17A. DHA, dihydroartemisinin.

**Figure 3.** DHA attenuates the inflammatory response of IL-17A-stimulated HaCaT cells. (a) The mRNA expression of TNF-α, IL-1β and IL-6 was detected by RT-qPCR; (b) The quantitative inflammatory factor assays including TNF-α, IL-1β and IL-6 were measured using ELISA kits; (c) Relative p-NF-κB p65/ NF-κB p65 expression was detected by Western blotting. ***P < 0.001 vs. control. ##P < 0.01 and ###P < 0.001 vs. IL-17A. DHA, dihydroartemisinin.

### DHA inhibits IL-17A-stimulated HaCaT cell over-proliferation by targeting FGFR1

FGFR1 was found to be a possible target of DHA action by Swiss Target Prediction database prediction. The results of mRNA and protein expression of FGFR1 revealed that FGFR1 expression was increased after IL-17A stimulation. In addition, FGFR1 expression was significantly inhibited after DHA intervention, including the most significant inhibition by 30 μM DHA (Figure 4a,b). To further investigate the target of DHA action, SUN11602 was added to study as an FGFR1 agonist. Results of cell viability and cell proliferation staining photographs showed that DHA significantly inhibited IL-17A-induced cell over-proliferation, but the inhibitory effect of DHA was significantly reversed after activation of FGFR1 by SUN11602 as an agonist (Figure 4c,d). On the other hand, the results for the expression of proliferation-related proteins showed that SUN11602 also reversed the inhibitory effect of DHA on Ki-67, CYCLIN D1 and c-Myc (Figure 4e).

**Figure 4.** DHA inhibits IL-17A-stimulated HaCaT cell over-proliferation by targeting FGFR1. The mRNA (a) and protein (b) expression of FGFR1 under the intervention of IL-17A and DHA were detected by RT-qPCR and Western blotting, respectively; (c) Cell viability following addition of FGFR1 agonist SUN11602 was detected by CCK-8; (d) Cell proliferation was detected with EDU staining; (e) Cell proliferation-related protein expression including Ki-67, cyclin D1 and c-Myc were analyzed by Western blotting. ***P < 0.001 vs. control. ##P < 0.01 and ###P < 0.001 vs. IL-17A. ^Δ^P<0.05, ^ΔΔ^P<0.01 and ^ΔΔΔ^P<0.001 vs. IL-17A+DHA. DHA, dihydroartemisinin; FGFR1, fibroblast growth factor receptor 1.

### DHA inhibits migration, induces differentiation and reduces inflammatory responses in IL-17A-stimulated HaCaT cells by targeting FGFR1

As consistent with the previous assays, wound healing and Western blotting were used to measure cell migration and differentiation, and RT-qPCR, ELISA and Western blotting were performed to detect cellular inflammatory responses. As shown in Figure 5, DHA could significantly inhibit cell migration rate and migration-related protein MMP2 and MMP9 expression, on the contrary, the addition of FGFR1 agonist reversed this inhibition (Figure 5a,b). In other side, DHA could promote IL-17A-induced cell differentiation, however, the differentiation-promoting effect of DHA was significantly repressed after the activation of FGFR1 (Figure 5c). In the result of inflammatory response, the mRNA expression and content of TNF-α, IL-1β and IL-6 inhibited by DHA were increased by SUN11602 (Figure 6a,b). And, the results of inflammation-associated protein p-NF-κB p65/ NF-κB p65 expression again showed that SUN11602 could reverse the inhibited inflammatory response by DHA (Figure 3c).

**Figure 5.** DHA inhibits migration and induces cell differentiation in IL-17A-stimulated HaCaT cells by targeting FGFR1. (a) Cell migration was detected by using wound healing; (b) Cell migration-related protein expressions were analyzed by Western blotting, including MMP2 and MMP9; (c) Cell differentiation-related protein expressions were analyzed by Western blotting, including keratin1, keratin 10, involucrin and filaggrin. ***P < 0.001 vs. control. ###P < 0.001 vs. IL-17A. ^Δ^P<0.05, ^ΔΔ^P<0.01 and ^ΔΔΔ^P<0.001 vs. IL-17A+DHA. DHA, dihydroartemisinin.

**Figure 6.** DHA attenuates the inflammatory response of IL-17A-stimulated HaCaT cells by targeting FGFR1. (a) The mRNA expression of TNF-α, IL-1β and IL-6 was detected by RT-qPCR; (b) The quantitative inflammatory factor assays including TNF-α, IL-1β and IL-6 were measured using ELISA kits; (c) Relative p-NF-κB p65/ NF-κB p65 expression was detected by Western blotting. ***P < 0.001 vs. control. ###P < 0.001 vs. IL-17A. ^Δ^P<0.05, ^ΔΔ^P<0.01 and ^ΔΔΔ^P<0.001 vs. IL-17A+DHA. DHA, dihydroartemisinin.

## Discussion

DHA is the main active product of artemisinin and its derivatives, which has anti-inflammatory effects and can be involved in autoimmune regulation of immune diseases [10]. It has been reported that DHA can significantly improve the symptoms of dextran sulfate sodium-induced inflammatory bowel diseases by regulating the expression of inflammation, cellular connectivity-related genes and intestinal flora [16]. The studies found that DHA had protective and therapeutic effects on lipopolysaccharide-induced acute lung injury by inhibiting NF-κB signaling pathway in an Nrf2-dependent manner [17]; and protected against dextran sulfate sodium-induced colitis by inhibiting PI3K/AKT and NF-κB signaling pathways [8]. These indicated that the inhibitory effect of DHA on inflammatory diseases through NF-KB pathway was present. In the present study, the protein expression of p-NF-κB p65/ NF-κB p65 in IL-7A-induced HaCaT cells was negatively correlated with the dose of DHA. Once again, it was demonstrated that DHA could inhibit the expression of NF-κB p65 signaling.

It is of interest that psoriasis is a chronic inflammatory skin disease, often combined with hypertension, diabetes and cardiovascular disease, and is the most common immune-mediated disease [18]. Furthermore, IL-17A is a member of the IL-17 cytokine family involved in the immune response to infectious agents and in the pathogenesis of inflammatory autoimmune diseases [19]. And psoriasis is characterized by a high expression of IL-17A and IL-17 F, which act on immune and nonimmune cell types and promote tissue inflammation [20,21]. In psoriatic injury, IL-17A is involved in neutrophil aggregation and the formation of epidermal micro abscesses [21]. Researchers have found that IL-17A, along with other Th17 cytokines, also upregulated the production of chemokines implicated in the pathogenesis of psoriasis [22]. Therefore, the use of IL-17A-induced cellular models for the study of psoriasis has important clinical implications. Meanwhile, in the current study, the IL-17A simulated cell model was investigated for epidermal keratin-forming cell injury (psoriasis).

The present study demonstrated that HaCaT cells exhibited excessive proliferation, an increased cell migration and inflammatory response, and a significant inhibition of cell differentiation after IL-17A stimulation. These results are consistent with the pathological features of psoriasis [23,24]. Subsequently, IL-17A-stimulated cell models were incubated and studied using high, medium and low concentrations of DHA. The experimental results revealed that DHA inhibited cell proliferation, migration and inflammatory response and promoted cell differentiation in IL-17A-induced HaCaT cells compared with the control group, and the effect was more pronounced with increasing doses of DHA. This shows that DHA has a significant effect on IL-17A-induced HaCaT cell model. To further investigate the mechanism of DHA on IL-17A-induced HaCaT, possible targets of DHA were predicted and analyzed with Swiss Target Prediction database. And FGFR1 was selected for subsequent studies through screening.

FGFR1 is a fibroblast growth factor receptor that is expressed by cells while providing co-stimulation to the cells. This type of receptor allows T cells to respond to fibroblast growth factors expressed in response to injury and inflammation [25]. Existing studies have reported that FGFR1 can suppress inflammatory responses by regulating the NF-κB signaling pathway [26,27]. Notably, David et al. found FGFR1 expression in dermatitis by a global transcriptome analysis [28]. To gain further confirmation that DHA targets FGFR1 for anti-inflammatory effects, SUN11602, as an FGFR1 agonist, was introduced into the study. Once again, the proliferation, migration, differentiation and inflammatory responses of IL-17A-induced HaCaT cells were analyzed and found that a series of changes produced by DHA on IL-17A-induced HaCaT cells, such as reducing proliferation, inhibiting migration, promoting differentiation and suppressing inflammatory responses, were disrupted after activation of FGF21 by SUN11602. In other words, SUN11602 reversed the effect of DHA on IL-17A-induced HaCaT cells. This suggests that DHA exerts anti-inflammatory effects by targeting FGFR1.

## Conclusion

This study successfully demonstrates that DHA targets FGFR1 to inhibit IL-17A-induced hyperproliferation and inflammatory response in HaCaT cells, and provides a new idea for the therapeutic study of inflammatory skin diseases such as psoriasis.

## Highlights

- Dihydroartemisinin inhibits IL-17A-stimulated hyperproliferation and migration and induces cell differentiation in HaCaT cells.
- Dihydroartemisinin reduces the inflammatory response of IL-17A-stimulated HaCaT cells.
- Dihydroartemisinin acts on IL-17A-induced keratinocytes by targeting FGFR1.

## References

[1] Langley RG, Krueger GG, Griffiths CE. Psoriasis: epidemiology, clinical features, and quality of life. Ann Rheum Dis. 2005 Mar;64(Suppl 2):ii18–23; discussion ii24-5.1570892810.1136/ard.2004.033217PMC1766861

[2] Boehncke WH, Schon MP. Psoriasis. Lancet. 2015 Sep 5;386(9997):983–994.2602558110.1016/S0140-6736(14)61909-7

[3] Gonzalez-Parra S, Dauden E. Psoriasis and depression: the role of inflammation. Actas Dermosifiliogr. 2019 Jan - Feb;110(1):12–19.3050975910.1016/j.ad.2018.05.009

[4] Ogawa E, Sato Y, Minagawa A, et al. Pathogenesis of psoriasis and development of treatment. J Dermatol. 2018 Mar;45(3):264–272.2922642210.1111/1346-8138.14139

[5] Armstrong AW, Read C. Pathophysiology, clinical presentation, and treatment of psoriasis: a review. JAMA. 2020 May 19;323(19):1945–1960.3242730710.1001/jama.2020.4006

[6] Lowes MA, Suarez-Farinas M, Krueger JG. Immunology of psoriasis. Annu Rev Immunol. 2014;32:227–255.2465529510.1146/annurev-immunol-032713-120225PMC4229247

[7] Furue M, Furue K, Tsuji G, et al. Interleukin-17A and keratinocytes in psoriasis. Int J Mol Sci. 2020 Feb 13;21(4):1275.10.3390/ijms21041275PMC707286832070069

[8] Li N, Sun W, Zhou X, et al. Dihydroartemisinin protects against dextran sulfate sodium-induced colitis in mice through inhibiting the PI3K/AKT and NF-kappaB signaling pathways. Biomed Res Int. 2019;2019:1415809.3178159110.1155/2019/1415809PMC6875009

[9] Fan M, Li Y, Yao C, et al. DC32, a dihydroartemisinin derivative, ameliorates collagen-induced arthritis through an Nrf2-p62-Keap1 feedback loop. Front Immunol. 2018;9:2762.3053870910.3389/fimmu.2018.02762PMC6277526

[10] Liu H, Tian Q, Ai X, et al. Dihydroartemisinin attenuates autoimmune thyroiditis by inhibiting the CXCR3/PI3K/AKT/NF-kappaB signaling pathway. Oncotarget. 2017 Dec 29;8(70):115028–115040.2938313910.18632/oncotarget.22854PMC5777751

[11] Chen Y, Yan Y, Liu H, et al. Dihydroartemisinin ameliorates psoriatic skin inflammation and its relapse by diminishing CD8(+) T-cell memory in wild-type and humanized mice. Theranostics. 2020;10(23):10466–10482.3292936010.7150/thno.45211PMC7482806

[12] Chen Y, Tao T, Wang W, et al. Dihydroartemisinin attenuated the symptoms of mice model of systemic lupus erythematosus by restoring the Treg/Th17 balance. Clin Exp Pharmacol Physiol. 2021 Apr;48(4):626–633.3346993610.1111/1440-1681.13461

[13] Yang B, Gao X, Sun Y, et al. Dihydroartemisinin alleviates high glucose-induced vascular smooth muscle cells proliferation and inflammation by depressing the miR-376b-3p/KLF15 pathway. Biochem Biophys Res Commun. 2020 Sep 24;530(3):574–580.3275331810.1016/j.bbrc.2020.07.095

[14] Tu J, Yin Z, Guo J, et al. Acitretin inhibits IL-17A-induced IL-36 expression in keratinocytes by down-regulating IkappaBzeta. Int Immunopharmacol. 2020 Feb;79:106045.3186391810.1016/j.intimp.2019.106045

[15] Livak KJ, Schmittgen TD. Analysis of relative gene expression data using real-time quantitative PCR and the 2(-Delta Delta C(T)) Method. Methods. 2001 Dec;25(4):402–408.1184660910.1006/meth.2001.1262

[16] Lei Z, Yang Y, Liu S, et al. Dihydroartemisinin ameliorates dextran sulfate sodium induced inflammatory bowel diseases in mice. Bioorg Chem. 2020 Jul;100:103915.3245038310.1016/j.bioorg.2020.103915

[17] Huang XT, Liu W, Zhou Y, et al. Dihydroartemisinin attenuates lipopolysaccharideinduced acute lung injury in mice by suppressing NFkappaB signaling in an Nrf2dependent manner. Int J Mol Med. 2019 Dec;44(6):2213–2222.3166112110.3892/ijmm.2019.4387PMC6844637

[18] Kamiya K, Kishimoto M, Sugai J, et al. Risk factors for the development of psoriasis. Int J Mol Sci. 2019 Sep 5;20(18):4347.10.3390/ijms20184347PMC676976231491865

[19] Brembilla NC, Senra L, Boehncke WH. The IL-17 family of cytokines in psoriasis: IL-17A and beyond. Front Immunol. 2018;9:1682.3012778110.3389/fimmu.2018.01682PMC6088173

[20] Garzorz-Stark N, Eyerich K. Psoriasis pathogenesis: keratinocytes are back in the spotlight. J Invest Dermatol. 2019 May;139(5):995–996.3101053010.1016/j.jid.2019.01.026

[21] Von Stebut E, Boehncke WH, Ghoreschi K, et al. IL-17A in psoriasis and beyond: cardiovascular and metabolic implications. Front Immunol. 2019;10:3096.3201014310.3389/fimmu.2019.03096PMC6974482

[22] Blauvelt A, Chiricozzi A. The immunologic role of IL-17 in psoriasis and psoriatic arthritis pathogenesis. Clin Rev Allergy Immunol. 2018 Dec;55(3):379–390.3010948110.1007/s12016-018-8702-3PMC6244934

[23] De Rosa G, Mignogna C. The histopathology of psoriasis. Reumatismo. 2007;59(Suppl 1):46–48.1782834310.4081/reumatismo.2007.1s.46

[24] Tomalin LE, Russell CB, Garcet S, et al. Short-term transcriptional response to IL-17 receptor-A antagonism in the treatment of psoriasis. J Allergy Clin Immunol. 2020 Mar;145(3):922–932.3188384510.1016/j.jaci.2019.10.041

[25] Byrd VM, Kilkenny DM, Dikov MM, et al. Fibroblast growth factor receptor-1 interacts with the T-cell receptor signalling pathway. Immunol Cell Biol. 2003 Dec;81(6):440–450.1463624110.1046/j.1440-1711.2003.01199.x

[26] Lai SW, Bamodu OA, Tsai WC, et al. The therapeutic targeting of the FGFR1/Src/NF-kappaB signaling axis inhibits pancreatic ductal adenocarcinoma stemness and oncogenicity. Clin Exp Metastasis. 2018 Oct;35(7):663–677.2998767110.1007/s10585-018-9919-5

[27] Tsubaki M, Takeda T, Matsuda T, et al. Activation of serum/glucocorticoid regulated Kinase 1/Nuclear Factor-kappaB pathway are correlated with low sensitivity to bortezomib and ixazomib in resistant multiple myeloma cells. Biomedicines. 2021 Jan 4;9(1):33.3340663910.3390/biomedicines9010033PMC7823718

[28] Ewald DA, Noda S, Oliva M, et al. Major differences between human atopic dermatitis and murine models, as determined by using global transcriptomic profiling. J Allergy Clin Immunol. 2017 Feb;139(2):562–571.2770267110.1016/j.jaci.2016.08.029

